# Adaptive Fluorodeoxyglucose-Positron Emission Tomography Based Chemotherapy Selection for Metastatic Non-small Cell Lung Cancer

**DOI:** 10.7759/cureus.18804

**Published:** 2021-10-15

**Authors:** Keith D Eaton, Perrin E Romine, Renato G Martins, Antoine Leblond, Laurie L Carr, Hubert J Vesselle

**Affiliations:** 1 Medical Oncology, University of Washington, Seattle, USA; 2 Nuclear Medicine, Centre Hospitalier de l'Université de Montréal (CHUM), Montreal, CAN; 3 Oncology, National Jewish Hospital, Denver, USA; 4 Nuclear Medicine, Fred Hutchinson Cancer Research Center, Seattle, USA

**Keywords:** paclitaxel, cisplatin, metastatic, adaptive clinical trial, (18f)-fdg pet, non-small cell lung cancer

## Abstract

Objectives

The change in tumor fluorodeoxyglucose (FDG) uptake by positron emission tomography (PET) scan after one cycle of platinum-based chemotherapy has been shown to predict progression-free and overall survival (PFS and OS) among advanced non-small cell lung cancer (NSCLC) patients. Using early FDG-PET response to determine subsequent chemotherapy, we aim to evaluate the role that adaptive chemotherapy regimens have on later CT response, PFS, and OS in patients with advanced NSCLC.

Materials and Methods

Chemotherapy-naïve patients with metastatic NSCLC received carboplatin and paclitaxel (CP) on day one and repeated FDG-PET on day 18. PET-responding patients continued CP chemotherapy for a total of four cycles. PET non-responders were switched to alternate docetaxel and gemcitabine (DG) for three additional cycles. The primary outcome was the CT Response Evaluation Criteria in Solid Tumors (RECIST 1.0) response. Secondary endpoints included PFS and OS.

Results

Forty-six patients initiated treatment with chemotherapy on trial and were evaluable by PET/CT. Of these, 19 (41%) met the FDG-PET criteria for the response after a single cycle of CP. Only one non-responding patient had a CT response. Despite the lack of CT response in the DG arm, no trend for worse PFS or OS was seen between the two arms.

Conclusions

This work demonstrates that changing chemotherapy in the event of non-response by PET did not lead to improved CT RECIST response. However, non-responding patients who switched chemotherapy had similar PFS and OS to those who responded by PET and continued the same regimen.

## Introduction

In clinical practice, CT is the predominant method for assessing the response to chemotherapy for solid tumors. This is based on data demonstrating that response by CT is a surrogate marker for improved predict progression-free (PFS), overall survival (OS), and quality of life (QOL) [1-3]. Response assessment by CT is limited by two factors: (1) Patients are typically assessed after several cycles of therapy, as the response by CT is gradual, and (2) CT is limited in the ability to differentiate slow tumor growth and a cytostatic effect of treatment. Lack of progression by CT referred to as the disease control rate has been shown to be the best CT predictor of survival in non-small cell lung cancer (NSCLC) [4].

As metabolic changes occur much earlier than tumor shrinkage in response to therapy, fluorodeoxyglucose-positron emission tomography (FDG-PET) has been investigated to assess the response early during cancer treatment [5-8]. The promise of adaptive therapy based on FDG-PET response has become the standard of care in the treatment of Hodgkin lymphoma [9]. Serial FDG-PET has been used successfully to predict early response in a variety of tumors including lymphoma [10,11], breast [12,13]. colorectal [14], esophageal [8,15], gastrointestinal stromal (GIST) [16], pancreas [17], ovarian [18], and lung cancer [19-23]. Increasing data points to the predictive role of FDG-PET imaging response in NSCLC treated with immunotherapy or tyrosine kinase inhibitors [24-28]. However, despite nearly two decades of study in solid tumors, there is insufficient data to support the widespread adoption of this strategy.

The first and most compelling study of FDG-PET for early response assessment in lung cancer was reported in 2003 [29,30]. This study demonstrated that FDG-PET response after one cycle of platinum-based chemotherapy in advanced NSCLC closely correlated with time to progression (TTP) and OS. Subsequent work [21-23,31] confirms these findings and suggests that FDG-PET is a powerful early biomarker for chemotherapy response in NSCLC independent of the chemotherapy regimen. Further work has demonstrated that early FDG-PET response can be used to guide subsequent treatment choices in resectable NSCLC, with an overall improvement in radiographic response [32]. This trial builds on these studies and tests the hypothesis that early response assessment by FDG-PET can be used to individualize the selection of chemotherapy in metastatic NSCLC. 

This study was conceived prior to the widespread adoption of current chemoimmunotherapy regimens for NSCLC. Carboplatin/paclitaxel was chosen as the initial doublet as this was the most commonly utilized therapy. Docetaxel/gemcitabine was chosen as the alternate regimen for metabolic non-responders (MR-) as there are two phase III trials showing overall survival that was not statistically different from the reference platinum doublet comparator arm [33,34]. Furthermore, there is evidence from a phase II study by Kosmas that patients previously treated with paclitaxel and a platinum agent respond to docetaxel/gemcitabine with a PR in 13/43 (33%) [35].

Given prior work demonstrating the predictive nature of early FDG-PET response, we hypothesize that outcomes from chemotherapy can be improved by determining early tumor response with FDG-PET and changing chemotherapy agents in the event of poor response by PET.

## Materials and methods

Study design

This is a single-center phase II trial accruing from 2007-2011. The study schema is presented in Figure 1. Enrolled patients underwent CT scan as well as baseline FDG-PET scan on day one prior to commencing cycle 1 of carboplatin with an area under a curve (AUC) equal to six and paclitaxel (175 mg/m2) chemotherapy. A repeat FDG-PET scan was done between days 18-21. Subsequent therapy was based on PET metabolic response; the response was defined prospectively as a decrease in standardized uptake value (SUV)max of ≥ 20% as prior work at our institution demonstrated a within-subject coefficient of variation in SUV of 10%. Metabolic responders (MR+) continued carboplatin/paclitaxel every 21 days for three additional cycles. Metabolic non-responders (MR-) were switched to gemcitabine (1000 mg/m2) on days one and eight, docetaxel (75 mg/m2) on day eight, and pegfilgrastim 6 mg subcutaneous (SQ) on day eight or nine every 21 days for the subsequent three cycles. The MR- subgroup underwent an additional PET/CT during cycle 2 between days 18-21. All patients were to complete four cycles of chemotherapy in total, with repeat FDG-PET/CT and CT scans done following completion of chemotherapy. This study was approved by the University of Washington IRB and was registered under the National Clinical Trial Registry (NCT00564733). Written consent was obtained at the time of study enrollment. 

**Figure 1:** Study Schema. PET: positron emission tomography; PC: paclitaxel/carboplatin; DG: docetaxel/gemcitabine; EOT: end-of-treatment.

Patient eligibility

Patients with histologically or cytologically confirmed NSCLC not amenable to curative intent therapy were eligible [American Joint Committee on Cancer (AJCC) 7th edition stage IIIB (pleural effusion) or stage IV]. Patients were required to have measurable disease, defined as at least one lesion that can be accurately measured in at least one dimension (> 10 mm with spiral CT scan) [36]. Patients were eligible if baseline FDG-PET scan demonstrated a target lesion with SUV > 3 that was ≥ 2 times the background uptake. Patients were excluded if they had received prior treatment with conventional cytotoxic chemotherapy for NSCLC but may have had prior radiotherapy or been treated with epidermal growth factor receptor (EGFR) tyrosine kinase inhibitors (TKI). One week must have elapsed after discontinuation of TKI prior to the initial PET scan. Patients who received radiotherapy must have recovered from the side effects of therapy (except alopecia) and have measurable disease outside of the radiation field. Other eligibility criteria included: age ≥ 18 years, life expectancy ≥ 3 months, Eastern Cooperative Oncology Group (ECOG) performance status 0-2, and adequate organ and marrow function.

(18F)-FDG PET imaging procedure

Initial and repeat imaging was performed using the same protocol on two cross-calibrated GE Discovery STE (DSTE) PET/CT systems (GE Medical Systems, Waukesha, WI). Patients fasted for 12 hours prior to injection of 10 mCi (370 MBq) (18F)-FDG administration. Blood glucose measurements were less than 150 mg/dL. A PET/CT from the base of the skull to mid-thigh was acquired in 2-D mode 60 minutes after the injection and reconstructed with random, scatter, and attenuation correction using the filtered back-projection algorithm (reconstruction parameters: 12 mm Hanning filter, 55 cm image diameter, 128 x 128 matrix). The CT scan was acquired using a low dose technique (60 mA, 0.8-sec tube rotation at 120 kVp).

Quantitative imaging analysis

For all patients, the analysis of PET scans was completed prior to response evaluation by CT. CT scan results were characterized per response evaluation criteria in solid tumors (RECIST) 1.0 criteria [36]. The PET target lesion used for calculation of ΔSUV was selected prospectively at the time of study entry by designated radiologists at the University of Washington Medical Center. This was the primary lung lesion if it had not been previously irradiated. In cases where there was no apparent primary lesion (e.g. relapse after surgery), the dominant metastatic lesion was used as the target lesion.

Primary outcome measures and statistical analysis

The primary outcome of this trial was the radiographic response by CT RECIST criteria following four cycles of chemotherapy. This study utilized response criteria based on the best response by the end of treatment. As this was an adaptive clinical trial, we hypothesized that changing chemotherapy would result in a response rate that is significantly better than the expected response rate of < 5% in this subpopulation if the initial carboplatin/paclitaxel therapy was continued.

To test this hypothesis, we planned to study 52 patients. Anticipating a dropout rate of 10% or less, we expected to have at least 45 patients complete at least one cycle of chemotherapy and have early response assessment by PET/CT. We compared the CT response rate in the initial metabolic non-responders to the observed response rate in metabolic non-responders in the work of Weber, which is 4% (1/27 patients). We expected N ≈ 20 initial non-responders by FDG-PET based on prior work demonstrating a 50% metabolic response rate following one cycle of cisplatin/paclitaxel (per prior work by Weber et al).

Using a predicted baseline response rate of p0=0.04, we defined a clinically interesting response rate as p1=0.2. A single sample test of proportions testing p1 > p0, using an exact calculation based on the binomial distribution, gives the power of 0.79 for a one-sided 0.05 level test. This would result in a positive trial if three or more patients out of the 20 responded. We justified the use of a one-sided test because the inferiority of the PET-based chemotherapy selection would not be clinically important to detect. Patients who were not evaluable were classified as non-responders. As such, this study has a simple criterion for success - observation of at least three responses as measured by CT at the end of four cycles of chemotherapy in the subset of patients who did not show evidence of response by PET to their initial chemotherapy with carboplatin/paclitaxel.

Secondary outcome measures

Secondary outcomes included PFS and OS. Additionally, this work sought to further validate previous work indicating that early PET is predictive of subsequent radiographic response [19,21-23,29,31,32]. Due to the intervention of changing therapy in initial non-responding patients, we could not directly verify these results. However, we could test corollary hypotheses in specific patient subsets, namely:

1) Initial metabolic responders to carboplatin/paclitaxel would have a high response rate by CT at the end of therapy,

2) Subsequent metabolic responders to docetaxel/gemcitabine would have a high response rate by CT at the end of therapy, and

3) Metabolic never responders would be unlikely to respond by CT at the end of therapy.

Among all patients who demonstrated an initial response to carboplatin/paclitaxel, we calculated the proportion of responders by CT at the end of therapy and compared these results directly to the proportion of metabolic responders in prior work [29]. Among patients who do not show metabolic response to carboplatin/paclitaxel and are subsequently treated with docetaxel/gemcitabine and demonstrate a metabolic response, we calculated the proportion of responders by CT at the end of therapy. We hypothesized that the CT response rate in the metabolic responders by a second response assessment by PET would be similar to that seen in metabolic responders to initial platinum doublet therapy. Among patients who showed no evidence of early metabolic response to either carboplatin/paclitaxel or subsequent docetaxel/gemcitabine, we calculated the proportion of non-responders by CT at the end of therapy. This subgroup was compared to the analogous subgroup of metabolic non-responders to initial platinum doublet therapy in the Weber series. Patients who withdrew from the study due to intolerance of chemotherapy, need for concomitant treatment, or symptomatic or radiographic progression prior to the final CT evaluation were classified as non-responders by CT and were included in the denominator of the above proportion.

## Results

Patient characteristics

In total, 55 patients consented to this trial. Four patients withdrew from the study prior to beginning treatment, and five were deemed ineligible following enrollment, with 46 undergoing treatment (Figure 2). Baseline patient characteristics are summarized in Table 1. Treatment was well tolerated, with no unexpected toxicities or adverse events. Treatment-related toxicities are summarized in Appendix 1.

**Figure 2:** CONSORT diagram. PET-CT: positron emission tomography-computed tomography; MR: metabolic response; EOT: end-of-treatment; PR: partial response; SD: stable disease; PD: progressive disease

**Table 1:** Demographic and baseline clinical characteristics NSCLC: non-small cell lung cancer; CNS: central nervous system; EGFR TKI: epidermal growth factor receptor tyrosine kinase inhibitors; ECOG PS: Eastern Cooperative Oncology Group Performance Status

N	All subjects (N=46)	MR+ (N=19)	MR- (N=27)
Median Age	62	64	58
Males	52%	47%	56%
Stage IIIB (pleural effusion)	11%	5%	15%
Stage IV	89%	95%	85%
Adenocarcinoma	65%	58%	70%
Squamous	24%	26%	22%
Other NSCLC	11%	16%	7%
Treated CNS metastases	28%	32%	26%
Prior EGFR TKI	9%	5%	11%
ECOG PS			
0	17%	21%	15%
1	76%	79%	74%
2	7%		11%

Radiographic and metabolic response

Of the initial 46 patients who underwent treatment, 19/46 (41%) were found to be initial MR+ and 27/46 (59%) were deemed to be MR-. Four of the MR- patients withdrew from the study (three due to progressive disease, one due to side effects), the remaining 23/46 were switched to docetaxel/gemcitabine (Figure 2). Eight out of 23 of the MR- patients treated with docetaxel/gemcitabine and three out of 19 of the MR+ patients continued on carboplatin/paclitaxel subsequently withdrew prior to completing four cycles of chemotherapy due to side effects and/or declining performance status. These patients are included in the progressive disease (PD) group for all further analysis. Of those patients initially classified as MR-, only one out of 27 patients was shown to have a radiographic response per RECIST criteria on CT scan following four cycles of chemotherapy. Of the initial MR- patients, however, 10/27 demonstrated stable disease on follow-up imaging after a total of four cycles of chemotherapy. Radiographic response stratified by the metabolic response for both this study population and the historic reference population described by Weber et al. is shown in Table 2. 

**Table 2:** Radiographic response at end of treatment stratified by metabolic response following cycle 1 for current study, cycle 2 for Weber study PR: partial response; SD: stable disease; PD: progressive disease

	MR+		MR-	
	Weber	Current	Weber	Current
% of patients	28/57 (49%)	19/46 (41%)	29/57 (51%)	27/46 (59%)
PR	20/28 (71%)	9/19 (47%)	1/29 (3%)	1/27 (4%)
SD	7/28 (25%)	6/19 (32%)	10/29 (34%)	10/27 (37%)
PD	1/28 (4%)	4/19 (21%)	18/29 (62%)	16/27 (59%)

Progression-free and overall survival

PFS and OS for both this study cohort and for the comparison cohort as described in Weber et al. are presented in Table 3. All study participants had over five years of follow-up with a median PFS of 125 days and OS of 265 days. Kaplan Meier OS and PFS curves for MR+ and MR- patients are presented in Figures 3, 4. The Weber work showed a statistically significant difference of over 100 days in PFS and OS between MR+ and MR- subjects. In contrast, the PFS for the MR+ (148d) and MR- (97d) were not statistically different (log-rank p=0.14). Also in contrast to the Weber data, we observed no difference in overall survival between the MR+ (273) and MR- (223) group (log-rank p = 0.43). 

**Table 3:** Median progression-free and overall survival MR+: Metabolic responders; MR-: metabolic non-responders P-values reflect published and calculated log-rank test values from respective Kaplan Meier Curves by Weber et al. and the current work. For current work, N=46 for all subjects, N=19 for MR+, and N=27 for MR-. For Weber et al., N=55 for all subjects, N=28 for MR+, and N=27 for MR-

	PFS (days)		OS (days)	
	Weber	Current	Weber	Current
All Subjects	143	125	222	265
MR+	163	148	252	273
MR-	54	97	151	223
P-value	0.0003	0.14	0.005	0.43

**Figure 3:** Kaplan-Meier overall survival curve censored at 5 years, stratified by metabolic response on Day 18 FDG PET imaging. Metabolic response was defined as ≥ 20% decrease in SUV of the dominant lesion.

**Figure 4:** Kaplan Meier progression-free survival curve censored at 5 years, stratified by metabolic response on Day 18 FDG PET imaging. Metabolic response was defined as ≥ 20% decrease in standardized uptake value of the dominant lesion.

## Discussion

Our hypothesis that changing chemotherapy in MR- patients would improve the CT-RECIST response rate after four cycles of chemotherapy was not confirmed. The secondary outcome measures did show that metabolic responding patients (MR+) were likely to respond by CT RECIST with a positive predictive value (PPV) of 47%, comparable to the PPV of 71% seen by Weber. This underscores the potential utility of early PET to predict subsequent CT response. Table 2 further highlights that among the current study’s MR- group, rates of PR, SD, and PD are similar to those seen in the Weber et al. study despite the alternative chemotherapy regimen that these patients received.

In contrast to other adaptive chemotherapy trials [32], a very low CT response rate was seen in the MR- patients who were switched to an alternative chemotherapy regimen (1/27, or 4% in the current trial as compared with 6/13, or 46%, in previously published work). There are many possible reasons for this difference, including the stage of the patients (metastatic vs. non-metastatic), sample size, and the alternative chemotherapy regimen that was used (docetaxel/gemcitabine vs. docetaxel/vinorelbine). Of patients who came off study after treatment initiation, 12 out of 15 were secondary to treatment-related toxicities, likely reflective of the regimen used, while only three were due to disease progression, and it is possible that this further impacted our results.

While our study failed to meet the primary endpoint, the adaptive treatment did not appear to be harmful, as the overall survival of our entire cohort was comparable to historic controls. In the Weber data, a sharp contrast was seen between the metabolic responders and non-responders, with a statistically significant difference in overall and progression-free survival of about 100 days. In our study, there was no statistically significant difference between the MR+ and MR- groups in PFS and OS.

It is important to acknowledge that the standard of care treatment for NSCLC has changed significantly since this study was conducted. There has been a paradigm shift away from conventional chemotherapy to immunotherapy and molecularly driven therapies. However, the therapeutic approach and study design utilized in this trial are still instructive, as there remains a strong case for developing tools to assess for predictive biomarkers and/or early response evaluation to avoid the toxicities and cost of ineffective treatments. FDG-PET markers have been shown to carry predictive and prognostic weight in patients with advanced NSCLC treated with immunotherapy and tyrosine kinase inhibitors, as well as in other solid tumors in the neoadjuvant setting [13,17,24-28,37-40]. Additionally, there are ongoing trials evaluating the use of adaptive-radiation therapy techniques based on interim FDG-PET response [41]. This work could potentially inform other efforts examining the use of PET as a surrogate marker for adaptive therapy response. Ultimately such an approach would need to be validated in randomized control trials in order to be incorporated into routine clinical care.

## Conclusions

In summary, this study failed to demonstrate a predictive CT response benefit by utilizing radiographic metabolic response following one cycle of cytotoxic chemotherapy to adapt further chemotherapy. However, OS and PFS were comparable between the metabolic responders and non-responders, suggesting a possible underlying survival benefit from the adaptive chemotherapy regimen. Response or disease control rate by CT remains an imperfect surrogate for the overall clinical benefit for patients with metastatic NSCLC. This study highlights that FDG-PET is a promising alternative surrogate, but there is insufficient data to adopt it in clinical practice for response assessment to palliative cytotoxic chemotherapy.

## Appendices

Appendix 1 

**Table 4:** Treatment-related toxicities N= 46; SAE: serious adverse event; *CTCAE version 3.0 used for grading AE’s; †Only grade 3 and higher adverse events or adverse events that led to a dose reduction or dose delay were captured. Hospitalizations related to disease progression were not captured as SAEs.

Adverse Event	All Grades*	Grade 2	Grade 3	Grade 4	SAE†
Thrombocytopenia	7 (15.2)	2 (4.4)	3 (6.5)	2 (4.4)	
Dyspnea	5 (10.9)		3 (6.5)	2 (4.4)	
Fatigue	5 (10.9)		4 (8.7)	1 (2.2)	
Pain (NOS)	5 (10.9)		5 (10.9)		
Anemia	4 (8.7)		3 (6.5)	1 (2.2)	
Neutropenia	3 (6.5)		1 (2.2)	2 (4.4)	1
Hypercalcemia	2 (4.4)	1 (2.2)		1 (2.2)	1
Leukopenia	2 (4.4)			2 (4.4)	
Pleural effusion	2 (4.4)	2 (4.4)			
Pneumonia	2 (4.4)		1 (2.2)	1 (2.2)	1
Tachycardia	2 (4.4)		2 (4.4)		
Acute renal insufficiency	1 (2.2)	1 (2.2)			1
Alanine aminotransferase (ALT) increased	1 (2.2)		1 (2.2)		
Anxiety	1 (2.2)		1 (2.2)		
Atelectasis	1 (2.2)			1 (2.2)	
Thromboembolic event	1 (2.2)		1 (2.2)		
Dehydration	1 (2.2)		1 (2.2)		
Fever	1 (2.2)	1 (2.2)			
Hypoalbuminemia	1 (2.2)		1 (2.2)		
Hypoxia	1 (2.2)		1 (2.2)		
Lymphocyte count decreased	1 (2.2)		1 (2.2)		
Nausea	1 (2.2)		1 (2.2)		
Sepsis	1 (2.2)		1 (2.2)		1
Syncope	1 (2.2)		1 (2.2)		
Vomiting	1 (2.2)		1 (2.2)		
